This article has been retracted.

# Research on Teaching Design of Geochemistry and Biology under the Background of Ecological Environment and Information Technology

**DOI:** 10.1155/2022/3785862

**Published:** 2022-04-21

**Authors:** Lei Jiang, Na Yu

**Affiliations:** College of Teacher Education, East China Normal University, 230061 Shanghai, China

## Abstract

The current social situation is that the rapid development of science and technology has brought about rapid economic growth, but the wanton development of ecological environmental resources, resulted in environmental deterioration, so that human survival faces major challenges. This is not only the current state of life but also an urgent problem that people will work together to solve. Therefore, in order to cultivate environmental awareness, make students intuitively and clearly understand the benign operation of ecological environment and the close relationship between people and the environment, this paper designs and studies the existing information technology to design biology teaching on the basis of the sustainable development of ecological environment and encourages students to strengthen the protection of the environment. This paper studied and designed the practical inquiry, analysis, and questionnaire survey. The experimental results show that the students in information technology teaching perform better than the traditional students, which can stimulate students' enthusiasm, arouse their interest in learning, and deepen students' understanding. The number of outstanding students increased by 5, and the number of failed students decreased by 8. The research significance of this paper is to provide new teaching design ideas for the existing biology teaching mode so that the development of information technology can benefit biology teaching.

## 1. Introduction

Ecological environment is the basis of human survival and life. Only when the ecological environment is well developed, can human beings be safe and guaranteed. However, the current ecological environment is not optimistic. Due to people's unreasonable development and utilization of nature, the balance of the ecosystem is destroyed, the ecological crisis is deepening, and the bad weather occurs frequently. In order to enable students to better understand the operation of nature and ecosystems, teaching biology with modern information technology is a good teaching method.

Currently, there are many studies on teaching design in the context of information technology. For example, Qianqian and Yao said that in the face of the current curriculum reform, information technology has been widely used in junior middle school teaching, and the combination of information technology and biology teaching has become the main trend in the development of biology teaching [1]. Yan Jiasheng said in relevant research that although high school biology accounts for only a small part of the college entrance examination results, it is also a very important high school course and plays a very important role in students' comprehensive scores [2]. Gao said that the deepening of the new technological revolution has promoted the application of information technology in the field of education, profoundly affected the process of classroom teaching reform in different disciplines, injected infinite vitality into the classroom, and promoted the overall improvement of classroom teaching quality [3]. Ye said that the development of modern information technology has gradually become an important auxiliary to the current teaching work. Using information technology to carry out teaching work can bring a new style to biology teaching and realize efficient classroom construction [4]. Therefore, the teaching design of biology under information technology is a research direction worth trying.

This paper begins with a simple understanding of the concept of ecological sustainable development and then studies the relevant knowledge and materials of information technology. Then, it explores and designs the network teaching platform, designs the teaching process, and studies the microcourse teaching and inquiry teaching methods under information technology. Finally, the conclusions were drawn by comparing the experiments and the questionnaires.

Interest is an important driving force to acquire knowledge, and the use of information technology to strengthen the intuition in the teaching process can not only attract students but also stimulate students' thirst for knowledge. Multimedia is used to show the microworld, macroscale the microcontent in biology, improve the teaching efficiency, and promote the effectiveness of teaching.

## 2. Biology Teaching Design Based on the Sustainable Development of Ecological Environment and Information Technology

### 2.1. Ecological Sustainable Development

#### 2.1.1. Development Evaluation

An ecosystem is mainly composed of several elements, such as nature, economy, and social life. The ecological quality evaluation indicators mainly involve resources, environment, and population, that is, the degree of resource surplus, environmental quality, and the living conditions of the population [5]. The selection of eco-environmental indicators is affected by topography and has diversity. For example, it can be evaluated from the aspects of biological abundance, vegetation coverage, water network density, social economy, environmental factors, ecosystem, road traffic, urban expansion, and ecological landscape pattern. In 2021, the Ministry of Ecology and Environment will incorporate the biodiversity index into the comprehensive evaluation index system of ecological quality.

#### 2.1.2. Ecological Environment Characteristics

  Global: environmental problems are widespread around the world, with some environmental problems such as greenhouse effects, ozone layer depletion, and acid rain. It has the most diverse influences and harms for the whole world and all mankind.
  Sociality: from the perspective of social life, ecological issues have covered all aspects of society [6].
  Political: the social nature of ecological problems will inevitably lead to political problems.
  Integrity: integrity means that the various components and elements of the ecological environment form a system [7, 8].
  Uncertainty: the so-called uncertainty refers to the inability to accurately predict the impact of current ecological problems on the future. The main reason for uncertainty lies in the limited knowledge and practical characteristics.
  Irreversibility: ecoenvironmental problems have irreversible characteristics, mainly manifested in the disappearance of resources and populations.

#### 2.1.3. Ecological and Environmental Issues

1. Ozone layer destruction: it is widely used in industrial, agricultural, and household sprays (chlorofluorocarbons for deodorants) and high-altitude aircraft, which are the killers of the ozone layer.
2. Acid rain: industrial production and the development of thermal power have greatly increased the emissions of air pollutants.
3. Land resources: soil depletion, soil degradation, soil erosion, and land salinization have become serious problems all over the world.
4. Natural resources: due to excessive deforestation, overgrazing of grasslands, and destruction of mountain tree planting, the desertified areas are expanding day by day.
5. Water resources: improper treatment of industrial and urban sewage pollutes rivers, lakes, and groundwater and further aggravates the severity of the freshwater resource shortage.
6. Mineral resources: the development and utilization of mineral resources caused serious damage and waste.
7. Air pollution: air pollution is mainly concentrated in cities, and coal and automobile exhaust are the main sources of pollution.
8. Waste pollution: the disposal volume of industrial solid waste and municipal waste is increasing.
9. Biodiversity is reduced: due to environmental degradation, the rate of biodiversity reduction is accelerating [9].

### 2.2. Information Technology

#### 2.2.1. The Status Quo of the Application of Information Technology in the Inquiry-Based Teaching of High-School Biology

At present, there are many research studies on the integration of information technology and courses, but relatively few research studies are related to biology. The content mainly involves the research of information technology in promoting the transformation of learning methods in biology teaching. The application of resources ignores the subject characteristics and operability [10].

#### 2.2.2. The Theoretical Basis of Information Technology and Curriculum Integration

The integration of information technology and curriculum serves teaching and learning, so it is inseparable from the theoretical basis of teaching and learning.

#### 2.2.3. The Significance of Information Technology and Curriculum Integration

The integration of information technology and curriculum is mainly designed to select the appropriate tools in the subject teaching. It can effectively organize and integrate the teaching content and promote the implementation of collaborative teaching strategies. In a computer-based interactive multimedia learning environment, students can choose the learning content suitable for their own level. At the same time, students can use multimedia to watch, listen, and operate manually. Students' independent learning cultivates students' ability to obtain information and grasp information and improves their interest in learning. At the same time, the information technology collaboration teaching strategy can give multiple learners the opportunity to observe, compare, analyze, and synthesize the same problems from different perspectives, in order to reflect [11, 12].

#### 2.2.4. Advantages

1. Teaching information is more abundant: information technology can be used to create a certain teaching situation with rich material resources, provide students with more various forms of materials and information, and help students understand the teaching content.
2. Independent study and independent development: students can use the communication methods provided by the online courseware to conduct independent exploration and research.
3. Convenient and economical: once the online course system has been constructed, in the subsequent use process, various inputs such as manpower and funds are relatively small.

### 2.3. Network Teaching Platform

Based on the demand results analyzed from the perspective of information ecology, the entire online education platform is designed with the information ecological balance as the entry point for the development of the online education platform. To build an online education platform, based on realistic teaching, to achieve resource sharing, it is necessary to focus on the internal architectural design of the online education platform.

The system design based on the evolution of the information ecology is mainly the opening of the system source code and the interfaceization of the production of online courses. The design idea of the entire platform is led by the “information man,” centered on the distribution and accumulation of information resources, using superior hardware facilities, and citing the internal framework of the concept of information ecology to build an information cycle system [13], as shown in Figure 1.

As a software project of an online education platform, its purpose is to achieve a more reasonable internal structure of the online education platform, more efficient use of resources, and closer communication and connection of information people. Therefore, in the whole system design process, we pay more attention to the design of logical flow. The logical structure is mainly divided into three major parts, namely the back-end management layer, the front-end display layer, and the database storage [14].

With the rise of the Internet, WEB technology has become more and more mature, and the B/S structure has emerged at the right time. Its basic working mode is that users access and share all information in server-side database storage with the client's browser. Its architecture mainly includes three major sections in Figure 2.

1. Configuration environment for system operation:
2. Server-side configuration environment requirements:
3. Operating system: WinXP/win2013 server
4. Database management system: SQL Server Web
5. Server: Microsoft IIS 6.0 and above
6. Hardware requirements: Intel (R) Celeron (R) 540 and above
7. Client configuration environment requirements:
8. Operating system: WinXP/win2003 server/Win7/Win8
9. Browser: Microsoft Internet Explorer 5.0 and above
10. Hardware requirements: Intel® Celeron® 430 and above

### 2.4. Teaching Design

#### 2.4.1. Meaning

Teaching design can arrange all kinds of teaching resources reasonably and effectively so that it can maximize the scientific, serialized, behavioral, artistic, and other effects. First, the instructional design highlights the subjective status of the students. Secondly, the teaching design can effectively control the teaching process. Third, teaching design can standardize teaching activities. Finally, teaching design can effectively improve teaching efficiency and teaching effect [15, 16].

#### 2.4.2. General Process

1. Learning demand analysis is the analysis of the gap between learners' knowledge, skills, emotional attitude, and current values and the educational goals set in the expectation. Learning content actually refers to the “recent development area,” that is, the part that shortens the gap between reality and expectations [17, 18].
2. The learning objectives involve the expected changes in knowledge, skills, emotional attitudes, and values brought by the learners through the content of the course.
3. The design of the teaching process is the “climax” of each link of the teaching design. After completing the positive analysis, the starting point, end point, and teaching strategy of teaching are determined, and in the process of teaching design, these various resources are made reasonable, orderly, and scientific, and services are provided for learners.
4. Teaching evaluation is to verify whether the teaching has reached the prescribed teaching goals. This paper evaluates the effect of biological teaching design based on information technology through the association rule algorithm.

People often express association rules in a common form *M*⇒*N* and measure the strength of association between *M* and *N* in association rules. Two indicators, support and confidence, need to be used.

Support (*M*⇒*N*) represents a subset of both *M* and *N* in the database. The formula can be expressed as follows:

(1) $$\begin{array}{c} \text{Support}\left(M\Rightarrow N\right)=\text{Support}\left(M\cup N\right)=Q\left(M\cup N\right). \end{array}$$

Confidence (*M*⇒*N*) is the proportion of transactions that contain both *M* and *N* to the transactions that contain *M*, expressed as follows:

(2) $$\begin{array}{c} \text{Confidence}\left(M\Rightarrow N\right)=\frac{\text{Support}\left(M\cup N\right)}{\text{Support}\left(M\cup N\right)}=Q\left(N|M\right). \end{array}$$

### 2.5. Problem-Oriented Teaching Design Supported by Information Technology

The problem design of problem-oriented teaching should follow the principle of “Trinity.” First, the teaching knowledge points in the teaching are to be reviewed and summarized, students should be allowed to edit and organize them through the screen, present them in the form of mind maps, and finally express their opinions.

In today's classroom teaching, PPT courseware has almost become one of the teaching aids that every teacher must use. Knowledge visualization is the application of visual representation of the creation and transmission of complex information between two or more people. The visual design principles of PPT courseware are as follows:

1. The characters are large and few. Facts show that students do not like to see slides with large sections of text, which prevents students from seeing the subject at a glance.
2. The format of this table is different from the picture, and the table is not as good as the picture. If you can use pictures to express information, try not to use tables. Using animation and video to convey information is better than using images.
3. Xuetong is not only suitable for online learning but also for offline classroom learning and training. It can organize and carry out various classroom activities. It can also learn, collect, count, and manage feedback and homework from students in each class.

### 2.6. Feasibility Analysis of the Application of Microclasses in Biology Teaching

1. Effectively improve the ability of students to learn independently: normally, if conditions permit, the school can allow students to use their mobile phones; then, teachers can set up a QQ group or Baidu network disk, make the knowledge points in the textbook into microclasses, and then pass them to the group file. Students can choose to watch microclasses according to their own situation and targeted learning.
2. Enriching classroom teaching methods: in biology classes, lectures, exercises, discussions, etc. are usually used. Of course, we will still use microclasses to teach. Microclasses mainly present teaching content in the form of video, with small limitations, strong practicability, and novel methods, which enrich the classroom teaching methods.
3. Obtain student feedback information in time: microclasses have the characteristics of “short,” “small,” and “precise,” and the teaching content is complete. At the same time, in terms of knowledge points that you do not understand, you can also focus on learning knowledge points you do not understand. You can solve problems by repeatedly watching microclasses or reading textbooks, and communicating with classmates and teachers.
4. Help students break through the key or difficult points of teaching: for novice teachers, there is not much teaching experience, and there are often situations where it is too late to complete the teaching task. Microclasses are just a breakthrough. Teachers can use microclasses to try to break through the difficult points of teaching and complete teaching tasks.

The teaching design plan is shown in Figure 3.

### 2.7. Construction of Inquiry Teaching Mode

#### 2.7.1. Selection and Characteristics of Biological Content

The selection of biological inquiry teaching content is divided into four categories: the first category is the basic concepts and rules that constitute the biological subject system; the second category is exploratory experiments; the third category is scientific issues in daily life that are closely related to the content of learning; the fourth category is scientific frontiers, social hotspot issues, and cross-disciplinary comprehensive issues.

#### 2.7.2. Mode Structure

The biological inquiry teaching mode under the information technology environment mainly includes the following five elements.

1. Combining the curriculum standards and actual teaching conditions appropriately determine the educational goals.
2. Teachers use multimedia tools, online teaching aids, virtual experiences, and other methods to show students the basic materials needed to explore new knowledge, create problem scenarios, and ask questions.
3. After guiding students into the situation, they should guide students to research and solve problems by themselves, encourage students to clarify their views through self-study and debate, actively feel in the process of meaning construction, and gain knowledge in the process of exploration.
4. Students and groups analyze and discuss in different ways, exchange their research results, and express research results in different ways. Teachers use multiple methods to evaluate all research activities.
5. After the teacher discovers the biological law through the exploration of a specific situation, he can extend it in a broad sense, guiding students to explore the biological law in a more general situation, thereby discovering the applicable conditions of the original law, and making the study more in-depth.

## 3. Questionnaire

### 3.1. The Purpose of the Experiment

Through experiments in biology classrooms, to understand what benefits the inquiry-based teaching model based on information technology will bring to students, the main purposes are as follows:

  Whether it can improve students' interest in biology;
  Whether it can improve students' ability to discover and solve problems;
  Whether it can improve students' innovative ability;
  Whether it can improve students' information literacy ability;

### 3.2. Scheme Design

This experiment is conducted using the controlled variable method. The experimental class is designed to compare with the control class. The experimental class uses information technology for biology teaching. The control class uses traditional teaching methods to learn. At the same time, it is necessary to maintain two classes of class hours, teaching content, and homework exercises. The content of the exam is the same.

### 3.3. Design of the Questionnaire

A questionnaire can have a more intuitive and clear understanding of the current situation, unify the different answers of questions for convenient analysis and comparison, and has a strong reference value. Therefore, this paper adopts the questionnaire method to investigate the learning effect of students after changing the teaching methods through information technology. The survey is designed in four aspects: whether students' learning attitude is improved; students' understanding of teaching content, and interest in biology courses are stimulated; and the impact of information technology on learning. These four aspects are used to understand the students' comprehensive learning situation.

### 3.4. Questionnaire Process

A total of 96 people were selected for this questionnaire, and they were divided into two groups. One group was a control group of 48 people who used traditional teaching methods to teach biology, and the other group was an experimental group of 48 people who used information technology to teach. A total of 100 questionnaires were issued, 96 of which have been filled out, and the effective response rate of the questionnaire was 96%. The questionnaire was followed up for one week.

## 4. Analysis of the Results of Biological Teaching Design of Information Technology

### 4.1. Biology Teaching Effect Supported by Information Technology

Regarding students' attitudes and teaching effects of using information technology to learn biology, the specific conditions are shown in Table 1.

As shown in Figure 4, interest in biology is still the most important learning factor, and the recognition of the role of information technology in teaching is also relatively high. Regarding the teaching content, more than half of the students believe that information technology makes the teaching content easier to understand and master.

### 4.2. Analysis of the Learning Effect of the Experimental Class and the Control Class on Biology

After a period of teaching, the teaching effect of the control class and the experimental class is based on the student's performance. The results show that the control class has 12 outstanding students who study in the traditional teaching method, and 10 people fail to learn through information technology. Of the people, the biological scores have improved significantly, 17 of them are excellent, and only 2 of them fail. The specific situation is shown in Table 2.

### 4.3. Emotional Attitude Analysis of Control Class and Experimental Class

The emotional attitude of this survey includes interest, recognition of scientific rigor, active independent participation, and good teamwork. In the control class, most people are interested in biology courses, followed by recognition of scientific rigor, and more people have a neutral view of cooperation. The specific situation is shown in Table 3.

As shown in Figure 5, students in the experimental class are most supportive of teamwork in biology class, followed by interest in biology class. Of course, compared with the control class, the experimental class is generally better than the control class in the four aspects of the investigation. Therefore, the use of information technology for teaching can better cultivate students' interest and learning ability in class.

## 5. Conclusion

The ecological environment advantages of cities with superior resource endowment are easier to be transformed into economic advantages, and the ecological environment is the basis of the sustainable and stable development of the economy and society [19]. Today, the frequent occurrence of extreme weather around the world makes us clearly realize that human beings will bear the consequences of the deterioration of the ecological environment. In this information age, we can not only keep an eye on changes in the global ecological environment and understand the symbiotic relationship between human beings and the environment but also use information-based methods to guide teaching and intuitively understand biology. We can use video and virtual technology to understand the laws of nature, study in-depth the basic operation of the ecosystem, and deepen the study of biology so as to understand the importance of protecting organisms and protecting the environment. The integration of information technology into biology teaching can more effectively improve the existing biology classroom teaching mode and deepen the influence of biology, which is undoubtedly a good medicine for teaching reform [20]. Through experimental research and investigation, it can be seen that the use of information technology for instructional design and curriculum development is a more effective way for students to learn and master knowledge points. Information technology not only improves students' attention and interest in learning but also deepens students' understanding of knowledge. Therefore, the use of modern technology in biology teaching means teaching can achieve twice the result with half the effort. Of course, the role of information technology in the education of other disciplines also needs further research and exploration.

## Figures and Tables

**Figure 1:** Information circulation system.

**Figure 2:** B/S architecture.

**Figure 3:** Biology instructional design process.

**Figure 4:** Biology teaching effect supported by information technology.

**Figure 5:** Emotional attitude analysis of experimental class.

**Table 1:** Biology teaching effect supported by information technology.

	Excellent	Good	Moderate	Poor
Learning attitude	23	12	6	7
Understanding of learning content	25	11	7	4
Interest	30	8	8	2
Impact	26	12	6	4

**Table 2:** Analysis of the learning effect of the experimental class and the control class on biology.

	Excellent	Good	Moderate	Poor
Control class	12	15	11	10
Experimental class	17	20	9	2

**Table 3:** Analysis of emotion and attitude of control class.

	Excellent	Good	Moderate	Poor
Interest	29	16	3	0
Scientific rigor	22	15	12	0
Autonomous participation	20	9	13	6
Like to cooperate	15	5	20	8

## Data Availability

The data underlying the results presented in the study are available within the manuscript.
